RETRACTED

# Motion Measurement and Analysis of Different Instruments for Single-Incision Laparoscopic Surgery

**DOI:** 10.1155/2022/3057485

**Published:** 2022-06-01

**Authors:** Kunyong Lyu, Lixiao Yang, Chengli Song

**Affiliations:** ^1^School of Information Science and Technology, ShanghaiTech University, Shanghai 201210, China; ^2^Equipment Department, Shanghai Changhai Hospital, Shanghai 200433, China; ^3^Shanghai Institute for Minimally Invasive Therapy, School of Health Science and Engineering, University of Shanghai for Science and Technology, Shanghai 200093, China

## Abstract

**Objective:**

To objectively compare and analyze the range of motion of three types of instruments for single-incision laparoscopic surgery. *Material and Methods*. Ten experienced participants were recruited. Straight instruments (Group A), straight/articulating instruments (Group B), and precurved instruments (Group C) were used to complete the transferring task through one site in a laparoscopic simulator. Straight instruments via two separate sites (Group D) served as control. The operation time of each group was recorded. Instrument positions were measured by an optical tracking system. The inserted length and pivoting angles were derived via MATLAB.

**Results:**

There was a significant difference in operation time between groups (D < A < B < C, *p* < 0.01). The range of motion of instruments was different on instrument types and surgical approaches. A significant difference in the inserted length was found between groups. Instrument conflicts and inadequate triangulation were found in Group A; instrument conflicts were found in Group B; no obvious conflicts and triangulation problems were observed in Group C. The operation in Group C was similar to the operation in Group D but differed on the left/right pivoting angles.

**Conclusion:**

Different types of instruments have different ranges of motion in single-incision laparoscopic surgery. Working with precurved instruments seems like a compromise to traditional laparoscopic surgery if the transmission property, and shaft curvature of the instruments could be improved. An integrated mechanical platform or robotic system might be the ultimate solution for single-incision laparoscopic surgery to pursue even less trauma.

## 1. Introduction

Single-incision laparoscopic surgery (SILS) is a potentially less-invasive technique compared with standard laparoscopic surgery (LAP) as it decreases the number of abdominal incisions. SILS is owned with many advantages, such as fewer scars, less trauma, shorter hospital stay, and fewer wound infections [1, 2]. However, the hypothesized advantages have not yet been proven thoroughly except its cosmetic effect [3]. In addition, several restrictions make SILS more difficult to learn and perform than LAP. Instrument conflicts and insufficient triangulation are inevitable because of the proximity and parallel entry of the working instruments through a single small incision [4–6].

RETRACTED

Two advanced instrumentations, articulating and precurved instruments, have been adopted for SILS to overcome the aforementioned restrictions. For straight and articulating instruments, cross-wise manipulation is often used to form effective triangulation; while for the precurved instrument, true-right and true-left manipulation is used, which can imitate the LAP approach and reduce mental workload. Various comparisons of performance have been done to find out which instrument of the three is most suitable for SILS. Manipulation method (cross or uncross) [7, 8] and instrument type [9, 10] through a single site have been compared and analyzed. The evaluation criteria include operation time [9], accuracy [8], electromyography [11], mental workload [7], and mechanical load [12]. However, instrument position has rarely been discussed and investigated in these studies. After all, it is the change of instrument location that leads to conflicts and inadequate triangulation in SILS. Position measurement and kinematic analysis of the instruments are a useful way not only to qualitatively understand the formation of conflicts and triangulation issues in SILS but also to quantitatively obtain the range of motion (ROM) and relative position of the instruments to the simulator. Studying the ROM of the laparoscopic instrument can help to determine the operation range inside the human abdomen and facilitate strategies for SILS, such as the innovative instrument design and surgical plan.

In general, several commercial tracking systems (electromagnetic, mechanical, and optical) are available to measure positions and movements. The feasibility of an optical tracking system for the measurement of the motion parameters was verified [13–16]. Studies show that the ROM of laparoscopic instruments is determined by surgical approaches, operation tasks, and left- or right-hand operation, while surgical experience is not viewed as a determining factor [14].

In this study, we utilize the optical tracking system MicronTracker, H3-60, to measure the ROM of the three most-used types of instruments via the SILS approach. Manipulation features of the three instruments are analyzed based on the movement and ROM of the instruments, and optimal configuration of the instrument for SILS is proposed.

## 2. Material and Methods

### 2.1. Apparatus and Setting

The tasks were performed with a laparoscopic simulator (SIMIT Scientific Co., Ltd., Shanghai, China), and the positions of the instrument during the operation were measured by an optical tracking system (MicronTracker®, H3-60, Claron Technology Inc., Toronto, Canada). Both LAP and SILS can be simulated with the multifunctional laparoscopic simulator (Figure 1(a)). Universal bearings were integrated into the insertion position of the simulator to guarantee the stability of the insertion point during instrument movement. Figure 1(c) shows the SILS access with two universal bearings.

RETRACTED

The optical tracking system (Figure 1(b)) works by identifying marks in the visible spectrum. Two types of the mark were designed. One is for the left instrument, and the other is for the right instrument. Fixation of the marks at the instrument handle (Figure 1(d)) did not interfere with the normal use of the instrument. Instrument positions were determined by the location of the marks and instrument tips, which can be recorded by the tracking system. Two straight graspers (Figure 2(a)) (SIMIT Scientific Co., Ltd., Shanghai, China), one articulating grasper (the instrument with the white handle in Figure 2(b)) (Cambridge Endoscopic Devices Inc., Framingham, MA, USA), and two precurved graspers (Figure 2(c)) (Olympus (China) Co., Ltd., Shanghai, China) were used to complete the tasks.

### 2.2. Tasks and Groups

Transferring task (Figure 3) was designed based on the basic tasks introduced by the Fundamentals of Laparoscopic Surgery program (SAGES/ACS, FLS program, Los Angeles, CA) [17]. Operators were required to transfer four rings from the left- to the right-side columns and then reverse the procedure to complete the task. Ten experienced participants were recruited, and all of them were naturally right-handed. Since surgical skill level is not a determining factor, the groups were not classified between participants. Groups were classified according to instrument type and approach: straight instruments via SILS (Group A), straight and articulating instruments via SILS (Group B), precurved instruments via SILS (Group C), and straight instruments via LAP (Group D, control) as shown in Figure 4.

### 2.3. Coordinate System on the Simulator

A coordinate system O*xyz* based on the simulator was established (Figure 5). Points A and B were the insertion points of the instruments on the simulator, which were the centers of the universal bearings, while Point C was the center of the task board. The middle point of A and B (O) was defined as the origin point. O→B was the positive direction of the *x*-axis, and O→C was the positive direction of the *z*-axis. The inserted length, pivoting angles, and relative position to the coordinate system of the instruments were calculated. The range was calculated as the difference between the maximum value and the minimum value.

RETRACTED

### 2.4. Procedure

Before the measurement, the mark templates and instrument tips were registered in the tracking system. Each participant performed Group D three times, then Group A three times, then Group B three times, and followed by Group C three times. Locations of the mark and instrument tip were recorded during the operation. Measurement results, including instrument position and reference points for the coordinate system, were imported into MATLAB R2015a (MathWorks, Inc., Natick, MA, USA) for data processing and analysis. The data were smoothed with a moving average filter (window length *n* = 3) at first, and ROM was then calculated. Operation time was also recorded, and a one-way analysis of variance (ANOVA) was used to investigate the difference in the completion time and ROM between groups. *p* < 0.05 was considered statistically significant.

## 3. Results

### 3.1. Operation Time

Figure 6 demonstrates the operation time and ROM of the instruments in each group. A significant difference was found in the time required to perform the task in different groups (D < A < B < C, *p* < 0.01). In SILS groups, operation time with the straight instruments (A) was the shortest, followed by the straight/articulating instruments (B) and precurved instruments (C), respectively. The accomplishment of tasks in LAP (D) took a shorter time compared with the SILS groups.

### 3.2. Range of Motion

As shown in Figure 6, the larger range of the inserted length was necessary to complete the task using the straight instrument (A) in comparison to the articulating (B) or precurved instruments (C). A significant difference was found (*p* < 0.05). The range of left/right pivoting angles between the three groups had no obvious difference, but a clear difference between the upper and lower limits could be noticed (Figure 6). The range of up/down pivoting angle of the straight instruments (A) was the largest, followed by the precurved instruments (C), and straight/articulating instruments (B), respectively.

Taking straight instruments in LAP (D) into consideration, the inserted length of the instruments in the LAP group was smaller than that in the SILS groups (*p* < 0.05). The range of pivoting angles in group D had no obvious difference compared to that in SILS. However, the upper and lower limits of the left/right pivoting angle of the instruments were quite different.

### 3.3. Instrument Position

Figures 7(a)–7(d) are the *xz* plane view of the position of the mark, insertion point, and instrument tip in Groups A, B, C, and D, respectively. From the *xz* plane view, left/right movement can be observed, and the left/right pivoting angles can be calculated in this plane. In Groups A, B, and C, the insertion points are close to each other (SILS), while in Group D, they are far from each other (LAP). Cross-wise manipulation was observed in Groups A and B. The tip of the left instrument is on the right side, and the tip of the right instrument is on the left side. In Groups C and D, true-right and true-left manipulations were used. The *xz* plane view also indicated the conditions of conflicts and triangulation. In Group A, there were two straight instruments, and the marks were located at the proximal end of the handle (Figure 2(a)). The location of the marks and tips indicated that instrument conflicts happened internally or externally. In Group B, there were straight and articulating instruments. The articulating instrument (dominant) was kept deflection at the distal tip, and there was a small pivoting angle at the handle as well. Therefore, instrument conflicts were not as severe as in Group A, but the cross-wise approach restricted the movement of the instruments, especially in the up-down direction. In Group C, there were precurved instruments, and true-right and true-left manipulations were used. It seemed that instrument clashes happened externally, but the location of the marks was on the proximal side of the shaft (Figure 2(c)). Handles were apart from each other due to the curved feature of the shaft. So, there were no handling conflicts. However, the straight portion of the instrument shaft was too long which caused slight conflicts between the left and right instruments. In Group D, there were two straight instruments in LAP. No instrument conflicts happened internally and externally, and true-right and true-left manipulations were adopted. Considering the profile of the instrument shaft and the *xz* plane view of the position, triangulation deficiency is obvious in Group A. In groups B and C, the triangulation problem was compensated by the curved profile of the instrument shaft, while in Group D, triangulation was compensated by the location of the insertion points.

RETRACTED

Figures 7(e)–7(h) are the *yz* plane view of the position of the mark, insertion point, and instrument tip in Groups A, B, C, and D, respectively. From the *yz* plane view, up/down movement can be observed, and the up/down pivoting angles can be calculated in this plane.

## 4. Discussion

The position of the insertion points in SILS is quite different compared to that in LAP, which is the main reason that causes a series of problems in SILS [4, 6]. In this study, a coordinate system was established based on the simulator, and then the ROM of three types of instruments in SILS and LAP was measured and analyzed. The position of the mark, instrument tip, and insertion points clearly showed the actual spatial position that the instrument could reach during operation. Considering the profile of the instrument shaft, it is easy to analyze the issue of instrument conflicts and triangulation. However, it is hard to draw a sound conclusion on which instrument is the best.

Straight instruments are most commonly used in clinics. Operation skills are accumulated during the long-term use of straight instruments either in the operation room or in the training, and even special tips have been developed. As expected, the operator spent less time with straight instruments to complete the transferring task in SILS than with the other two types of instruments, although instrument conflicts and triangulation problems were the most severe during the three. Familiarity with the tools is an important factor for the operation time. The introduction of the articulating instrument in Group B abated the triangulation constraints to some extent, and cross-wise manipulation was still used. Bending of the instrument tip and handle during the operation facilitated the use and measurement of the instrument. Although triangulation was easily formed compared to the straight instruments, operation time with the straight and articulating instruments was longer than that with the straight instruments alone, which is in accordance with the results in [10, 18].

The precurved instrument is a recent development in the instrumentation of SILS. The shaft of the instrument is rigid with at least one curved segment. In this study, double-curved instruments from Olympus were used. Theoretically, instrument conflicts and cross-wise manner could be avoided, and triangulation could be easily formed. Measurement results indicated that a cross-wise manner was avoided indeed, and triangulation was easily formed as well [19]. The ROM and operation manner were similar to the straight instruments in LAP. But operation time using precurved instruments was the longest. There were several reasons. First, although there are two curved segments in the instrument shaft, the straight part of the instrument is too long that the middle part of the instrument works like the straight instruments. Instruments conflicted internally if the inserted length increases or conflicted externally if the inserted length decreases. Second, the transmission property of the precurved instrument is a problem. Due to the friction inside the instrument shaft, opening or closing the jaws is awkward and might cause severe aches to the hands. In addition, rotation of the tip always lagged with the rotation of the knob at the handle. And this might cause misoperation because of the inaccurate transmission. Third, as analyzed above, the precurved instrument is new to the operator, and familiarity plays an important role here.

RETRACTED

Among the three types of instruments, the precurved instrument works most similar to the traditional LAP operation [19] and has the potential to be well used for SILS if the curvature of the shaft and transmission property could be improved. However, with the pursuit of even less trauma in SILS, the incision size at the umbilicus will be even smaller. Instrument conflicts will be inevitable by using these handheld instruments. Integrated mechanical platforms [20, 21] or robotics [22, 23] might be the ultimate solution for SILS. Among these integrated systems, there are no pivoting points at the insertion point anymore. The ROM is also a key parameter to consider when developing or evaluating these kinds of systems.

This study was based in a dry laboratory, and a built-in camera was used instead of the laparoscope. Thus, conflicts between instruments and laparoscope could not be simulated. Operation position and insertion points of the instrument with simulator were ideally set up. Only one transferring task was tested. Further complex tasks or clinical investigations should be carried out to confirm the effect of instrument types in different settings.

In conclusion, this study introduced a method to measure the ROM of laparoscopic instruments during an operation. Different types of instruments have different ranges of motion in SILS. Working with the precurved instrument in SILS can avoid instrument conflicts and insufficient triangulation and seems like a compromise to LAP if the transmission property and shaft curvature of the instrument could be improved. An integrated mechanical platform or robotic system might be the ultimate solution for SILS to pursue even less trauma.

## Figures and Tables

**Figure 1:** Apparatus and setting. (a) Laparoscopic simulator. (b) Tracking system. (c) SILS access with universal bearings. (d) An instrument with tracking marks.

**Figure 2:** Location of the marks in the instruments. (a) Straight instruments. (b) Straight and articulating instruments. (c) Precurved instruments.

**Figure 3:** Transferring task. In this image, the straight instruments via LAP (Group D) are illustrated.

**Figure 4:** The schematic diagrams of the four groups of ABCD. (a) Group A, two straight instruments via SILS. (b) Group B, one straight instrument and one articulated instrument via SILS. (c) Group C, two precurved instruments via SILS. (d) Group D, two straight instruments via LAP.

RETRACTED

**Figure 5:** Coordinate system on the simulator.

**Figure 6:** Operation time and ROM of instruments. Group A, straight instruments SILS; Group B, straight/articulating instruments SILS; Group C, precurved instruments SILS; Group D, straight instruments LAP. ^∗^Significant difference was found between groups in the operation time and interested length. *p* < 0.05.

**Figure 7:** Position of the mark, insertion point, and instrument tip. (a–d) The *xz* plane view of instrument position in Groups A, B, C, and D. (e–h) The *yz* plane view of instrument position in Groups A, B, C, and D (red points: left instrument; black points: right instrument). The middle point of A and B (O) was defined as the origin point. O→B was the positive direction of the *x*-axis, and O→C was the positive direction of the *z*-axis as shown in Figure 5.

## Data Availability

The data used to support the findings of this study are included within the article. If some researchers need more detailed data, it will be available from the corresponding authors upon request.
